The article "Prevalence and public health significance of rabies virus in bats in the North Region of Cameroon" was retracted in 2024. Reasons: unreliable results or conclusions; concerns about the data; concerns about the results or conclusions.

# Prevalence and public health significance of rabies virus in bats in the North Region of Cameroon

**DOI:** 10.1371/journal.pntd.0010803

**Published:** 2023-10-23

**Authors:** Isaac Dah, Rodrigue Simonet Poueme Namegni, Mohamed Moctar Mouiche Mouliom, Simon Dickmu Jumbo, Ranyl Nguena Guefack Noumedem, Isabelle Conclois, Liegeois Florian, Laurent God-Yang, Jean Marc Kameni Feussom, Abel Wade, Dorothée Missé, Julius Awah-Ndukum

**Affiliations:** 1 School of Veterinary Medicine and Sciences, The University of Ngaoundéré, Ngaoundéré, Cameroon; 2 National Veterinary Laboratory (LANAVET), Garoua, Cameroon; 3 MIVEGEC, IRD, Univ. Montpellier, CNRS, Montpellier, France; 4 University of Zimbabwe, Faculty of Veterinary Science, Harare, Zimbabwe; 5 Epidemiology-Public Health-Veterinary Association (ESPV), Yaoundé, Cameroon; 6 Cameroon Epidemiological Network for Animal Diseases (RESCAM), Ministry of Livestock, Fisheries and Animal Industries (MINEPIA), Yaoundé, Cameroon; 7 Department of Animal Science, Faculty of Agronomy and Agricultural Sciences, University of Dschang, Dschang, Cameroon; 8 Department of Animal Production Technology, College of Technology, University of Bamenda, Bambili, Cameroon; Addis Ababa University, ETHIOPIA

## Abstract

**Background:**

Rabies is a zoonotic disease of all warm-blooded animals including humans. There is a paucity of data on the status of rabies in wild animals in Cameroon and the disease is endemic in the country with dogs being the main source of transmission. Bat habitats are widespread in Cameroon, but there is limited information on the prevalence of rabies in bats, and their role of as potential reservoirs of rabies virus.

**Methods:**

A cross sectional study was carried out to estimate the prevalence and to assess risk factors of rabies virus in bats in the North Region of Cameroon. A total of 212 bats belonging to three families (Pteropodidae, Vespertilionidae and Molossidae) and 5 species were sampled in 7 localities in the North Region of Cameroon and were tested for rabies virus antigen using direct Immunofluorescence Test (IFA).

**Results:**

Overall, 26.9% (57/212) of the bats collected showed an IFA positive reaction. The prevalence was significantly higher (P<0.05) in adult bats (33.3% (36/108)) compared to young individuals (20.2%; 21/104). The main risk factors identified in the study for human exposure to bats were gender (Male), religion (Christianity), localities (Babla and Lagdo), the practice of bat hunting, bat consumption, unawareness of bat rabies and cohabitation with bats in close proximity.

**Conclusion:**

The study revealed the first evidence of Lyssavirus in bats in Cameroon. This finding showed that bat rabies are real and represents a potential public health concern in communities with bat habitats in the North Region of Cameroon. Enhancing the level of public awareness and health education on the potential of bats as reservoirs of Lyssavirus in Cameroon as well as the integration of the “One Health” approach for effective management of animal and human rabies should be emphasized.

The article "Prevalence and public health significance of rabies virus in bats in the North Region of Cameroon" was retracted in 2024. Reasons: unreliable results or conclusions; concerns about the data; concerns about the results or conclusions.

## Author summary

Rabies is a zoonotic disease caused by a virus of the genus Lyssavirus. It affects all warm-blooded animals including humans. Canine and human rabies are well documented as endemic in Cameroon, but little is known about this disease in wildlife, in particular among bats, despite their multiple interactions with the inhabitants of North Region of Cameroon. Indeed, bats are hunted, sold and consumed as bush meat by the local populations. We investigated the presence of Lyssavirus in bats and assessed the risk factors of human exposure to bats in the North Region of Cameroon. The study highlights that the rabies virus is present in bats in this area. The population was aware of human and canine rabies, however, the presence of the disease in bats was less known. Based on these findings, investigating bat populations on a large scale, to characterise the rabies virus circulating in the region, as well as educate the local population on the risks factors of rabies transmission from bats to humans and other animals are strongly recommended.

## Introduction

Rabies is a virulent fatal zoonotic disease of major public health concern caused by a Lyssavirus [1]. The virus is known to affect all warm-blooded animals, including domestic pets, which are the main vectors. Bat Lyssaviruses are distributed worldwide including canine rabies-free countries and bats are the primary dispensers of Lyssavirus to other animals and humans over vast geographical areas through their saliva and urine [2]. Bats have been directly involved in the transmission of rabies to humans through aerosols and unapparent bites as well as indirectly through animals they infected Infections of others animal could be through contact with contaminated body fluids by scratching of mucous membranes and open skin wounds [3–7]. Fatalities in humans and other animal species due to bat Lyssavirus [8–10], as well as human rabies related to bat Lyssavirus variants, have been reported to be associated with bat biting and simple contact with bats [11]. Bat Lyssaviruses are more infectious in superficial epidermal inoculation and multiply faster in non-nerve cells at a lower temperature than the canine rabies virus [12]. The transmission of animal rabies to humans is higher in areas where animal rabies is widespread [13], and there are frequent human and animal exposures to bats, including sick and injured bats with high risk of contamination [14].

The article "Prevalence and public health significance of rabies virus in bats in the North Region of Cameroon" was retracted in 2024. Reasons: unreliable results or conclusions; concerns about the data; concerns about the results or conclusions.

Rabies has induced over 3.7 million disability-adjusted life years (DALYs), with 8.6 billion USD in economic losses annually and 59,000 human deaths per year worldwide [15]. Bat Lyssavirus could be underestimated in Africa, due to insufficient surveillance programs [16]. The disease has been reported in bat populations in parts of the continent with prevalence ranging from 29 to 67% in Kenya [17], 38% in Ghana [18], 19% in Nigeria [19]) and 5.5% in the Democratic Republic of Congo [20]. In Cameroon, over 576,232.88 USD was estimated as direct financial losses linked to rabies prevention measures and post-exposure treatments between 2004 and 2013 in three cities (Garoua, Yaoundé and Ngaoundéré) of Cameroon [21]. Urban rabies is widespread in dogs, which are considered as the main source of animal and human rabies in Cameroon [21–25] and canine and human rabies are endemic in the North Region of the country [21,23,26]. There are many bat colonies and a majority of bat roosting sites are located adjacent to human communities where the level of physical interactions between bats and humans is high in many parts of the country. However, there is little or no information on the epidemiology of bat Lyssaviruses. Insectivorous bats frequently flock and inhabit roof-tops and homes while hunting of frugivorous bats for food is common in Cameroon. According to Mickleburgh *et al*. [27], the consumption of these animals by local populations could endanger the long-term survival of these species (*Eidolon helvum)*. Indeed, *E*, *helvum* is consumed and marketed locally in the Bomboko area (South-West) and elsewhere in Cameroon, where they constitute an important source of income for local hunters [27]. In addition, human–wildlife interactions that increase the risk of transmission are frequent and various, namely hunting, butchering and consumption of wild animals, including bats, are common in Cameroon [28]. Additionally, subsistence activities and large-scale agriculture expose people not only to bat bites, but to potential infection through scratching due to the presence of urine and droppings of bats [28]. In the North Region of Cameroon, bats usually form colonies in the roofs, trees and abandoned tall structures in human communities and are also hunted as a source of animal protein and their guano, is widely collected as fertilizer [29]. In this context, the present study was carried out to estimate the prevalence of rabies virus in bats and to assess the associated risk factors to human health in the Northern region of Cameroon to increase knowledge of the potential sources of rabies virus. This could contribute to the achievement of the global goal of rabies elimination by 2030.

The article "Prevalence and public health significance of rabies virus in bats in the North Region of Cameroon" was retracted in 2024. Reasons: unreliable results or conclusions; concerns about the data; concerns about the results or conclusions.

## Material and methods

### Ethic statements

Risk assessments of the project were performed by the researchers to avoid hazards to all persons involved in the study. To the best of our knowledge, apart from risk of stress and time wastage, participants were not exposed to any other risk related to this study. The scientific research and ethics committee of the School of Veterinary Medicine and Sciences of the University of Ngaoundéré provided ethical approval (007/2017/UN/ESMV/DAACRS/SSFC) for the study. Administrative authorizations were also obtained from the Regional Delegation of Wildlife and protected areas (ref: N°140/L/MINFOF/DRN/SRFAP) and the Governor of the North region (ref: N°195/AE/D/SG/DAAJ). The purpose, objectives and procedure of the study were explained to the participants. They were also informed that their personal data will be coded to respect anonymity. Besides they were informed that they are free to accept or refuse to participate to the study without any coercion. An oral consent was obtained from each participant prior to interview. For those less than 21 years old, the oral consent to participate was obtained from their parents or guardians

### Description of study areas

This study was carried out in 7 localities (Babla, Djalingo, Lagdo, Guider, Mayo Oulo, Yelwa and Garoua II) in two Administrative Divisions (Mayo-Louti and Bénoué) of the North Region of Cameroon (6° - 10° N and 12° - 16°E) (Fig 1) based on the available information on bat roosts, bat colonies and field observations of flying and foraging bats. The North Region is located in the Sudano-sahelian region with an average altitude of 249 m, a short rainy season from mid-March to October of 1200–1600 mm per annum and an ambient temperature range from 21° to 36°C.

**Fig 1:** Map showing study sites. Bats specimen were collected in several study sites (red stars) in Mayo-Louti and Bénoué administrative divisions of the North Region of Cameroon. Adapted source from DIVA-GIS: https://www.diva-gis.org/gdata; License: https://en.wikipedia.org/wiki/DIVA-GIS.

### Study design and sampling

A cross sectional study was conducted in the North Region of Cameroon from February to May 2017 following identification and listing of communities and geographical areas with bats roosts and bat activities. Information on bat roosts were obtained through the aid of leaders of the local communities. All identified localities with bat activities (hunting, selling of bat as bush meat etc.) were included and visited for sample collection during the study period. Insectivorous bats and Fruit bats were collected twice weekly from the hunters before delivery to their clients. Indeed, there were vendors who bought bats and resold the meat to the consumers in these localities. Summarily, 205 live bats and 7 dead bats (6 *Eidolon helvum* from the Garoua zoological garden and one *Chaerephon pumilus* from Lagdo) were collected. A total sample of 212 bats were studied, 76 frugivorous bats (*Eidolon helvum*) and 136 insectivorous bats (10 *Chaerephon chapini;* 10 *Chaerephon leucogaster;* 96 *Chaerephon pumilus* and 20 *Scotophilus leucogaster*).

The article "Prevalence and public health significance of rabies virus in bats in the North Region of Cameroon" was retracted in 2024. Reasons: unreliable results or conclusions; concerns about the data; concerns about the results or conclusions.

Whole animals were shipped to the National Veterinary Laboratory (LANAVET) Garoua in individual ziplock bag placed in a cooler with frozen ice packs [30]. A minimum sample size of 212 was determined according to Thrusfield [31].

### Bat identification

The bat species were identified based on biomorphometric measurements with calliper using dichotomous keys [29]. The gender of bats was determined based on the observation of external genital organs and stage of growth (whether the bats were juvenile or adult) was through appraisal of body development and pelage coloration as previously described [19,32].

### Laboratory analysis

Laboratory analysis was done at LANAVET Garoua, in the North Region of Cameroon.

### Direct immunofluorescence assay

A cross-section of the brain (including cerebral cortex and cerebellum) of each bats collected (212) in the study was taken after skull dissection in a certified biosafety cabinet [33]. An equal portion of each brain part collected was mixed and a thin smear spread on a slide was made. The slides were fixed in cold acetone at -20°C for one hour and then dried for 30 min at room temperature. The Lyssavirus ribo-nucleoprotein complex was detected using Rabies specific labelled polyclonal antibodies with Evans blue (1/2000 final dilution) as counterstain to denote stained areas and incubated at 37°C in a humidified chamber according to the manufacturer’s instructions. The direct Immunofluorescence Assay (IFA) was used to detect Lyssavirus antigen in brain tissue, in accordance with WOAH (World Organization for Animal Health) and WHO (World Health Organisation) recommendations [34].

Briefly, positive and negative canine rabies controls available at the National Veterinary Laboratory in Garoua were used to validate the test results. A test was validated when there was fluorescence in the positive control and no fluorescence in the negative control. Three experienced staff members read the test slides before validating the results. In case of discordance between the results of the three technicians, samples were retested and submitted blindly for lecture. In case of any discordance, we considered the results from the majorities (2/3).

The article "Prevalence and public health significance of rabies virus in bats in the North Region of Cameroon" was retracted in 2024. Reasons: unreliable results or conclusions; concerns about the data; concerns about the results or conclusions.

### Exposure assessment and questionnaire survey

To determine the risk factors of human exposure to bat, a structured questionnaire (S1 Text) was issued to 535 willing inhabitants around the bat collection sites. The households within 5km radius of the bats collection sites were randomly surveyed by simple number generation without replacement. The verbal consent of each respondent was obtained in advance to participate in the study. The consent to participate in the study for young responders (< 21 years old) was obtained from their parents or guardians. Each participant was interviewed individually to avoid communication bias during the survey. The questionnaire was structured to collect information on a range of variables including lifestyle, socio-demographic data, knowledge about rabies, bat activities and human–bat interactions.

### Data management and analysis

Data obtained in the study were entered into Microsoft Excel (Microsoft, PC/Windows XP, 2010, Redmond WA, USA) for descriptive statistics and transferred to IBM Statistical Package for Social Sciences Software (SPSS Inc., Chicago IL, USA) version 21 for further analysis. Simple logistical regression was used to assess the potential risk factors with their respective odds ratios and 95% confidence intervals [35]. Variables with p< 0.2 from the univariate analysis were included in a multivariate analysis to construct the best model based on the lower value of Akaike Information Criterion (AIC). Three models were constructed with the same dependent variable (exposure to bat). We have used as inputs in the first model canine and bat rabies awareness and their zoonotic aspect. In the second, the independent variables were the socio demographic characteristics of the respondents (religion, gender, occupation, level of education localities). The third model used as independent variables, human interaction with bats (presence of bat in the localities, in the home, bat hunting and bat consumption). As the dependent variable of all three models is the same (exposure to bats), we built the final model using the significant risk factors from each one. Exposure to bats was defined as having been bitten by a bat, scratched by a bat or touched a bat with bare hands [35,36]. The Khi-2 test or Fischer test were used to assess the association between the intrinsic and extrinsic characteristic of bats and bat rabies, between the knowledge and socio demographic characteristics of respondents. We considered the respondent has a good knowledge or was aware of rabies when he or she has heard about rabies, he or she knows that dogs and/or cats are the main vectors and knows that its manifestation in both dogs and humans include aggressiveness and mortality.

The article "Prevalence and public health significance of rabies virus in bats in the North Region of Cameroon" was retracted in 2024. Reasons: unreliable results or conclusions; concerns about the data; concerns about the results or conclusions.

## Results

### Prevalence of rabies in bats

Fifty seven (57) out of 212 (26.9%) bat brain samples were tested positive for rabies antigen using direct Immunofluorescence Assay (IFA) (Fig 2).

**Fig 2:** Detection of Rabies’ ribo-nucleoprotein complex using Direct Immunofluorescence Assay. Negative **(A)** and Positive **(B)** brain samples were fixed, analysed for the presence of the Rabies virus antigen and visualized under a fluorescence microscope (100X objective). Arrows indicate viral ribo-nucleoprotein complex.

### Human risk exposure to bat rabies

The proportion of respondents who were unaware of bat rabies were significantly 13.9 times more exposed to these flying mammals (Table 1) than those who didn’t answer to this question considered as reference.

**Table 1:** Univariate and multivariate analysis of risk factors of bat exposure according to respondent’s awareness on bat rabies and canine rabies in the North Region of Cameroon from February to May 2017.

Variables/ modalities	N (%)	OR (95% CI)	P	Global p-value	aOR (95%CI)	P
**Awareness to canine rabies**						
No	136 (38.2)	Ref	-	-	Ref	
Yes	399 (49.6)	1.6 (1.1–2.4)	0.02*	-	4.8 (0.6–40.3)	0.14
**Awareness to bat rabies**						
No	372 (49.5)	3.1 (1.3–7.6)	0.01*	<0.01*	13.9 (1.5–130.2)	0.02*
Yes	25 (64.0)	1.7 (1.2–2.6)	<0.01*		7.9 (0.9–66.2)	0.05
No response	138 (36.2)	Ref	-		Ref	
**Awareness to human transmission of Canine rabies**						
No	55 (50.9)	1.7 (0.8–3.1)	0.11	0.07	-	
Yes	342 (49,4)	1.6 (1.0–2.3)	0.03*		-	
No response	138 (38.4)	Ref			-	
**Awareness to human transmission of bat rabies**						
No	10 (40.0)	2.7 (0.6–12.0)	0.20	0.19	-	
Yes	25 (64.0)	1.3 (0.4–4.6)	0.71		-	
No response	500 (46.0)	Ref	-		-	

OR: odd ratio; aOR: adjusted odd ratio; CI: confidence interval; N: number of answers to specific question, (%) proportion of exposed respondents, Ref: reference, P: value

The study showed that more respondents were aware of canine rabies (74.6%, 399/535) than bat rabies (4.7%, 25/535). The level of awareness increased significantly with the level of education (Table 2). Male participants were significantly more informed about canine rabies than female participants.

**Table 2:** Proportion of respondents according to their knowledge on canine rabies and bat rabies with respect to their socio-demographic characteristics in the North Region of Cameroon (n = 535).

	Canine Rabies		Bat rabies	
Variables/modalities	N (%)	P-value	N (%)	P-value
**Localities**				
Babla	87 (6)	0.85	6 (6.9)	0.69
Djalingo	62 (74.2)		4 (6.4)	
Garoua II	70 (75.7)		2 (2.9	
Guider	107 (71.9)		6 (5.6)	
Lagdo	70 (78.7)		1 (1.4)	
Mayo Oulo	78 (71.8)		3 (3.8)	
Yelwa	61(80.3)		3 (4.9)	
**Age (years)**		0.07		0.42
15 – 25	203 (67.9)		7 (3.4)	
26 – 35	134 (76.1)		8 (5.9)	
36 – 45	92 (80.4)		5 (5.4)	
46 – 55	48 (77.1)		4 (8.3)	
56 – 65	58 (82.8)		1 (1.7)	
**Religion**				
Christians	348 (75.9)	0.59	21 (6.0)	0.05
Muslims	158 (72.8)		2 (1.3)	
Without religion	29 (68.9)		2 (6.9)	
**Gender**				
Female	209 (69.8)	0.04*	6 (2.9)	0.11
Male	326 (77.6)		19 (5.8)	
**Educational level**				
None	136 (66.9)	<0.01*	2 (1.5)	<0.01*
Primary	151 (73.5)		3 (1.9)	
Secondary	218 (77.1)		15 (6.9)	
Tertiary	30 (96.7)		5 (16.7)	
**Total**	**535 (74.6)**		**25 (4.7)**	

N: number of participants

*: p<0.05; (%): proportion of respondents who were aware of rabies in canine or in bats.

The article "Prevalence and public health significance of rabies virus in bats in the North Region of Cameroon" was retracted in 2024. Reasons: unreliable results or conclusions; concerns about the data; concerns about the results or conclusions.

The gender and religion of respondents influenced significantly (P<0.05) the level of exposure to bats in the North Region of Cameroon (Table 3). Males and Christians were respectively 2.9 times each more likely to be exposed to bats than female respondents and those without religion (Table 3). The final model explained significantly (64.5%) the observed effect.

**Table 3:** Univariate and multivariate analysis highlighting the risk factors associated with human exposure to bats in the North Region of Cameroon according to socio demographic characteristics of respondents from February to May 2017.

Variables/modalities	N (%)	Global P value	OR (95% CI)	P	aOR (95%CI)	P
**Gender**						
Male	326 (56.1)		2.7 (1.9–3.9)	<0,01*	2.9 (1.9–4.4)	<0,01*
Female	209 (32.1)		Ref		Ref	
**Age (years)**						
15–25	203 (50.1)	0.55	1.5 (0.9–2.5)		-	
26–35	134 (46.3)		1.3 (0.7–2.2)		-	
56–65	58 (46.5)		1.3 (0.7–2.5)		-	
46–55	48 (43.7)		1.1 (0.6–2.3)		-	
36–45	92 (40.2)		Ref		-	
**Educational level**						
Secondary	218 (54.1)	0.02*	1.9 (1.3–3.0)	<0,01*	-	
Tertiary	30 (50.0)		1.7 (0.7–3.7)	0.21	-	
Primary	151 (43.7)		1.3 (0.8–2.1)	0.29	-	
None	136 (37.5)		Ref		-	
**Religion**						
Christianity	348 (55.7)	<0.01*	2.9 (2.0–4.4)	0.01*	2.9 (1.6–7.1)	0.01*
Atheists	29 (31.0)		1.1 (0.4–2.5)	0.88	1.8 (0.6–4.6)	0.22
Islam	158 (29.7)		Ref		Ref	
**Occupation**						
Without occupation	17 (52.9)	<0.01*	1.7 (0.6–4.3)	0.34	-	
Scholars	143 (58.0)		1.9 (1.3–2.9)	< 0.01*	-	
Public workers	61 (47.5)		1.3 (0.7–2.2)	0.35	-	
Private workers	314 (41.1)		Ref		-	

N: number of participants, (%): proportion of respondents exposed to bat, CI: confidence interval

*: p ≤ 0.05. Ref: reference, OR: odd ratio, aOR: adjusted odd ratio

Additionally, among respondents who lived in proximity with bats 57.3% (306/535) reported that bats could be found in different places including the roof of bedrooms (24.1%; 129/535), trees (14.2%; 76/535), abandoned buildings (2.2%; 12/535) and warehouses (2.1%; 11/535). The following tools were used for bat hunting: sticks (66%; 353/535), chemical products (15.3%; 82/535), bare hands (9.3%; 50/535) and others (9.3%; 50/535) such as nets, sling, thorn, dress. According to them, the reasons for hunting the bats were due to their nuisance (69.0%; 356/535), for consumption (12.5%; 67/535), playing with bats (10.1%; 54/535), sociocultural practice (2.9%; 16/535), leisure (3.6%; 19/535) and research (1.8%, 10/535). Though some respondents (17.6%; 94/535) reported being bitten and scratched by bat during hunting, but none of them was vaccinated against rabies and none sought rabies post exposure prophylactic measures.

The article "Prevalence and public health significance of rabies virus in bats in the North Region of Cameroon" was retracted in 2024. Reasons: unreliable results or conclusions; concerns about the data; concerns about the results or conclusions.

The presence of bats in the localities and homes, bat consumption and bat hunting significantly (P<0.05) exposed respondents to bats. The respondents who have bats in trees and bedrooms, who hunted and ate bats, and who live in Lagdo and Babla localities were more likely to be exposed to bats (Table 4). The final model explained significantly (72%) the observed effect.

**Table 4:** Univariate and multivariate analysis of risk factors associated to bat exposure according to human interaction with bats in the North region from to February to May 2017.

Variables/modalities	N (%)	Global p-value	OR (95%CI)	P-	aOR (95%CI)	P
**Presence of bats in the home**						
Without bat in the home	307 (39.4)	<0.01*	0.4 (0.2–0.6)	<0.01*	0.4 (0.2–0.8)	< 0,01*
In abandoned room	12 (41.7)		0.4 (0.1–1.4)	0.17	0.2 (0.1–0.9)	0.04*
Store room	11 (18.2)		0.1 (0.03–0.6)	0.01*	0.1 (0.02–0.6)	0.01*
Bedroom	129 (57.4)		0.8 (0.4–1.4)	0.41	0.6 (0.2–1.1)	0.08
Trees in the house	76 (63.2)		Ref		Ref	
**Bats hunting**						
No	385 (37.1)		0.2 (0.2–0.4)	<0.01*	0.2 (0.1–0.4)	< 0,01**
Yes	150 (71.3)		Ref		Ref	
**Bats consumption**						
No	482 (40.8)		8.5.10^−9^ (8.510^−9^–8.6.10−^9^)	<0.01*	< 0,01	< 0,01*
Yes	53 (100)		Ref		Ref	
**Localities**						
Djalingo	62 (64.5)	<0.01*	7.4 (3.3–16.8)	<0.01*	1.9 (0.9–4.3)	0.81
Lagdo	70 (62.9)		6.9 (3.1–15.3)	<0.01*	2.6 (1.1–5.9)	0.02*
Babla	87 (58.6)		5.8 (2.7–12.4)	<0.01*	3.7 (1.6–8.7)	0.00*
Garoua II	70 (50.0)		4.1 (1.9–8.9)	<0.01*	1.7 (0.8–3.7)	0.18
Mayo Oulo	77 (42.9)		3.1 (1.4–6.6)	<0.01*	0.8 (0.4–1.6)	0.53
Guider	108 (32.4)		1.9 (0.9–4.1)	<0.09	0.4 (0.2–1.1)	0.06
Yelwa	61 (19.7		Ref		Ref	

N: number of participants, CI: confidence interval, (%): proportion of respondents exposed to bat

*: p ≤ 0.05. Ref: reference.

A higher risk of bat exposure was observed among the Christians (aOR: 3.1); male respondents (aOR: 2.6), bats hunters and those living in Djalingo (aOR: 3.0), Lagdo (aOR: 2.4) and Babla (aOR: 3.7) (Table 5). The final model registered the lower AIC value (185.3) than the three first ones and explained 74% of observed effects.

The article "Prevalence and public health significance of rabies virus in bats in the North Region of Cameroon" was retracted in 2024. Reasons: unreliable results or conclusions; concerns about the data; concerns about the results or conclusions.

**Table 5:** Final model of risk factors associated to bat exposure in the North region from to February to May 2017.

Variables /modalities	Coefficient	P-value	Adjusted OR (95% CI)
**Religion**			
Christianity	1.118	0.02*	3.1 (1.2–8.2)
Atheists	0.894	0.09	2.4 (0.8–6.9)
Islam			Ref
**Respondent’s gender**			
Male	0.963	<0.01*	2.6 (1.7–4.1)
Female			Ref
**Bat hunting**			
No	-1.491	< 0.01	0.2 (0.1-.0.4)
Yes			Ref
**Localities**			
Djalingo	1.101	0.01*	3.0 (1.3–6.9)
Lagdo	0.864	0.04*	2.4 (1.0–5.5)
Babla	1.304	< 0.01*	3.7 (1.5–8.9)
Garoua II	0.576	0.15	1.8 (0.8–3.8)
Mayo Oulo	-0.001	0.99	0.9 (0.5–2.1)
Guider	-0.002	0.73	0.7 (0.2–1.8)
Yelwa	-	-	Ref

*: p ≤ 0.05. Ref: reference, CI: confidence interval, Ref: reference

## Discussion

The present study reports the first evidence of Lyssavirus in bats in Cameroon and revealed rabies antigens in apparently healthy bats. This observation underline a potential risk for human communities living in contact with bats. The overall rabies prevalence (26.9%) might reflect the status of rabies in these animals although it could be due to sampling bias. Though we considered that bats in the population had an equal chance of being captured, it is possible that weak and unhealthy bats could have been captured more easily, which might have introduced a selection bias. It should be noted, however, that the majority of bats collected had a body condition score of medium to good. The prevalence of rabies recorded in the present study is lower than serological prevalence reported among vampire bats (*Desmodus rotundus*) (50.34%) in Brazil [37], in colonies of *Eidolon helvum* (40 to 67%) and *Roussetus aegyptiacus* (29 to 46%) in Kenya [17] and bat colonies (up to 59.3%) in Spain [38].

The findings of the present study are similar to those observed in moribund vampire bats (*Desmodus rotundus*) tested by IFA and PCR in northern Brazil [39]. The active infection has been reported in apparently healthy (0.1%) and moribund bats (9%) in other studies [17,40]. The prevalence of rabies virus in this study was higher than values reported among bat species in the United States (9% to 10%) [40] Canada (7%) [36] Spain (3.3 to 10%) [38], Nigeria (19%) [19] and Kenya (9%) [17]. The difference in infections rates may be associated with the method and period of sample collection during the dry season which is characterized by food scarcity, elevated temperature and peak infection of rabies in bat populations as reported by Pedro et al. [41], It is also interesting to note that Nigeria is a neighboring country of Cameroon bordered by the study area, and bat colonies in both countries could move from one country to the next and mix during their foraging. Indeed, *E*. *helvum* may travel hundreds of kilometers during certain season given the possibility to these bats to move from one roost to another [19]. The influence of season on the occurrence of rabies in bats such as higher rates during the dry season [41] and fluctuating and cyclical rabies infection in bat populations have been reported elsewhere [40]. The immigration of rabid bats into a colony can cause rapid spread of the infection through bites of infected bats during mutual grooming, mating and aggressive behaviour such as protection of the territory [42]. Indeed, unfavourable living conditions (climate, food source, immunity, density of the colony, parasite load among others), sex, age and physical depletion caused by stress, co-infections, sexual exhaustion and migration are major risk factors for rabies infection [10,17,38,40]. Salmon-Mulanovich et al [43] associated a higher prevalence of rabies in male bats with more aggressive behaviour (territory protection, defence against intrusion, fighting, and licking of body fluids during the breeding season). However, a high or similar prevalence of Lyssavirus in female bats than in males has been associated with gregarious maternity behaviour during hibernation [44]. In the present study, young bats were less likely to be infected with rabies virus than adults and older bats. Indeed, adult and older bats were more exposed due to their usual aggressiveness and adventurous behaviours and longer periods spent in the colonies. Adults could have been in continuous or intermittent contact with other bats in the same or in other colonies (some of which could have been infected) compare to young and juvenile bats. However, serological prevalence can be influenced by antibodies of maternal origin and bats exposed to the virus confer lasting immunity (6 to 8 weeks) in their offspring by placental and mammary routes [40].

The article "Prevalence and public health significance of rabies virus in bats in the North Region of Cameroon" was retracted in 2024. Reasons: unreliable results or conclusions; concerns about the data; concerns about the results or conclusions.

Due to a technical problem impacting samples conservation (RNA degradation) the molecular part of this work was not performed and represents a limitation to this study. It would be important to carry out an in-depth molecular study to identify with precision the Lyssavirus circulating in the region. This would help to understand the epidemiological pattern of Lyssavirus and identify potential reservoirs in Northern Cameroon. Overall, the findings of this study agree with those of Salmon–Mulanovich *et al*. [43] in Peru, Kuzmin *et al*. [17] in Kenya and Dzikwi *et al*. [19] in Nigeria who reported that the location of the bats does not influence the rabies infection rates in bats contrary to Costa *et al*. [45] who observed significant variations of bat Lyssavirus rates according to location. The difference was associated with sampling biases such as disparities in distances between location sites of bat populations and number of bats sampled at the different study sites. Given the vast temporospatial spread of the activities of bat colonies, bat populations in close locations (less than 100km apart) will have common features since they frequently mix and interact together and could be considered as the same colony. This is the case in the present study as Northern Cameroon borders Nigeria. The zoonotic transmission of bat Lyssavirus is well documented. Bat rabies can be transmitted to humans and other mammals over long periods and vast geographical areas through various routes including aerosols, unapparent bites and contamination of nerve tissue with saliva, urine and other body fluids of infected bats [2–7]. Based on the public health perception on bat rabies, respondents in rural localities around Garoua who shared the same environments with colonies of bats were more aware of canine and human rabies than of bat rabies. The finding was less than that observed by Bouli *et al*. [21] who recorded over 88.7% of rabies awareness levels in urban Garoua areas among respondents who were more literate and with better educational levels compared to those in rural areas. However, Moran *et al*. [35] reported that over 91% of the respondents living in the rural areas harbouring bat populations in Guatemala had little or no knowledge of rabies. Also, Costa and Fernandes [46] observed a strong positive correlation between educational levels and knowledge about rabies as reported in the present study.

Though the awareness about canine rabies was significantly relevant, most respondents seem to be ignorant of the zoonotic transmission potentials of bat Lyssavirus. Bouli *et al*., [21] recorded a lower bat rabies awareness level (0.3%) in communities of Garoua-Cameroon while higher levels ranging from 10%– 42% had been reported in Thailand and Guatemala due to widespread public awareness campaigns against rabies in these countries [35,47]. Similar to the level of knowledge about canine rabies recorded in the present study, the levels of awareness about bat rabies was significantly associated with literacy and educational level of the respondents. This finding highlights the ignorance of the communities about the potential risk of bats rabies and its transmission to other species including humans. Awah-Ndukum et al., [23] reported that dogs and cats were the main source and transmitters of rabies in Cameroon probably due to the common and visible manifestations of the disease in these species. The clinical manifestations of rabies are more furious and lethal in dogs [3] and non-lethal in bats [14]. The furious forms of rabies in dog usually constitute a canine rabies outbreak alert for human communities. Indeed, canine and human rabies is endemic in Cameroon, [21,23]. This may contribute to the better awareness of respondents on canine rabies than bat rabies. In the present study, the gender and educational level of respondents significantly influenced the levels of awareness of bat rabies.

The article "Prevalence and public health significance of rabies virus in bats in the North Region of Cameroon" was retracted in 2024. Reasons: unreliable results or conclusions; concerns about the data; concerns about the results or conclusions.

The presence of bats in the localities and homes, bat hunting and consumption, the gender and religion of respondents and localities may increase the risk of human exposure to bats. Having bats in the home may increase the probability of hunting them due to their nuisance or for consumption. Consumption of bats was frequent in the study communities in agreement with Kamins *et al*. [48] who reported that bat consumption was a cultural and food habit in Ghana. This habit to hunt and consume bats as meat and source of animal protein among communities explains the difference in level of exposure observed in the present study between gender and religious groups in favour of male and Christians. Indeed, some of the respondents reported that touching or consuming bats is strictly forbidden by Islam. Although the questionnaire used in the present study is very precise, we cannot rule out the possible human memory bias. Indeed, if exposure to bats is not a recent event, when answering the questions people may have forgotten if they have been bitten by a bat, scratched by a bat or touched a bat with bare hand. This memory bias in human survey could be overcome by a larger number of participants in the study.

## Conclusion

Rabies is a zoonotic disease of all warm-blooded animals including man. Though the disease is endemic in Cameroon, with dogs being the main source and transmitters. Bat habitats are widespread in many Cameroon environments. Bats usually form colonies in the roofs, trees and abandoned tall buidings in human communities and they are hunted as source of animal protein in the North Region of Cameroon. The present study has revealed a bat rabies prevalence of 26.9% and reports the first evidence of rabies in apparently healthy bats in the North Region of Cameroon. This finding could constitute a public health concern in communities living in proximity with bats in the North Region of Cameroon as well as bordering countries, such as Nigeria. Further large scale studies on bats should be undertaken in order to isolate and characterize the Lyssavirus circulating in the bat population in Cameroon. Public awareness campaigns and health education are essential to develop protective measures against rabies and understand the potential role of bats as reservoirs of rabies especially among human communities where bat colonies are found. It is important to note that, when bats were tested positive for Lyssavirus, people living near the study sites were informed and advised to visit a health care center. However, a major problem for the follow-up of people exposed to bats is that in the absence of clinical signs, they do not consult a clinician. This point demonstrates the need for joint multidisciplinary studies with clinicians that could lead to more effective human and animal surveys of this zoonotic disease. The study highlights the importance of investigating the dynamic of rabies virus transmission among animals and humans in this region and other parts of the country and to characterise the Lyssavirus type circulating among these flying mammals in Cameroon. Multi-sectorial sensitization of communities in the country to improve their level of awareness on bat rabies and integration of the “One Health” approach for effective management of rabies in Cameroon should be emphasized.

The article "Prevalence and public health significance of rabies virus in bats in the North Region of Cameroon" was retracted in 2024. Reasons: unreliable results or conclusions; concerns about the data; concerns about the results or conclusions.

## Supporting information

S1 Text Questionnaire survey. (PDF)
